RETRACTED

# A Classroom Emotion Recognition Model Based on a Convolutional Neural Network Speech Emotion Algorithm

**DOI:** 10.1155/2022/9563877

**Published:** 2022-07-07

**Authors:** Qinying Yuan

**Affiliations:** Xi'an Jiaotong University, Xi'an, Shaanxi 710049, China

## Abstract

In this paper, we construct a model of convolutional neural network speech emotion algorithm, analyze the classroom identified by the neural network with a certain degree of confidence together with the school used in the dataset, find the characteristics and rules of teachers' control of classroom emotion nowadays using big data, find the parts of classroom emotion, and design a classroom emotion recognition model based on convolutional neural network speech emotion algorithm according to these characteristics. This paper will investigate the factors and patterns of teachers' emotional control in the classroom. In this paper, the existing neural network is adapted and improved, and some preprocessing is performed on the current dataset to train the network. The network used in this paper is a combination of convolutional neural network (CNN) and recurrent neural network (RNN), which takes advantage of both CNN for feature extraction and RNN for memory capability in the sequence model. This network has a good effect on both object labeling and speech recognition. For the problem of extracting emotion features of whole-sentence speech, we propose an attention mechanism-based emotion recognition algorithm for variable-length speech and design a spatiotemporal attention module for the speech emotion algorithm and a convolutional channel attention module for the CNN network to reduce the contribution of the spatiotemporal data of the speech emotion algorithm and the unimportant parts of the CNN convolutional channel feature data in the subsequent recognition by the attention mechanism. In turn, the weight of core key data and features is increased to improve the model recognition accuracy.

## 1. Introduction

As CNN is applied in the speech domain and shows excellent performance, researchers have started to study the effectiveness of CNN in learning emotional features in speech signals, and many CNN-RNN-based frameworks for speech emotion recognition have been proposed. However, many emotion recognition problems are still waiting to be solved. We still do not know what kind of network is the most suitable and what feature extraction method can get the most compelling feature representation [1]. The accuracy of the SER system will directly affect whether the human-computer interaction can be completed smoothly, which is the key to making human-computer interaction more natural. The research of deep learning-based speech emotion recognition algorithm can firstly extract more effective speech emotion features by using the advantage of machine learning in feature extraction and improving the SER system's accuracy in recognizing emotions [2]. Second, a model with lower complexity means lower latency in recognizing emotions. Studying the complexity of the algorithm model and proposing methods to reduce the complexity of the model can effectively reduce the latency of the SER system, thus obtaining a better human-computer interaction experience. Therefore, we hope to propose a neural network model that is more suitable for emotion recognition and can better extract the emotional features in speech, resulting in higher accuracy and lower latency of emotion recognition.

RETRACTED

The human brain has a compelling information processing capability, which can perceive and understand the part of the information in a speech where the audio reflects the speaker's emotion; therefore, they can sense the change in the speaker's sentiment in address. As the most direct and effective way for people to communicate and transmit information daily, speech contains textual and acoustic data [3]. Auditory information refers to the characteristics the human ear can perceive, such as timbre, tone quality, volume, and rhythm of people's speech. Since the acoustic features corresponding to different emotional addresses have apparent differences, mathematical calculation methods are usually used to map the speech signal into the elements related to its emotion [4]. The computer can recognize the sentiment expressed by a speech. So far, research on speech emotion recognition has mainly used two methods: traditional machine learning and deep learning. Commonly used machine learning methods include hidden Markov model (HMM), K proximity algorithm, support vector machine (SVM), and Bayesian algorithm; as the development of machine learning algorithms becomes more and more mature, how to make machines think like human brains and make behavioral feedback becomes the focus of more and more scholars' research, which is also the point of deep learning research [5]. Deep learning mainly simulates how the human brain processes information by building multilayer neural networks, combining feature representation with knowledge, and creating a model through continuous learning. Commonly used deep learning methods are convolutional neural networks (CNN) for spatial data and recurrent neural networks (RNN) for time series data.

Emotions are the attitudes and experiences of human beings after comparing objective things with their own needs, which are closely related to human production life and have a vital role in human decision-making, interaction, and cognitive process [6]. For the current classroom emotion recognition research, firstly, there are relatively few relevant studies; most of the classroom emotion recognition research is based on visual, speech, text, behavior, physiological signals, and other modalities, among which visual and behavioral data such as facial expressions and body movements are complicated to capture and collect, and physiological signal data are not only challenging but also expensive to manage; secondly, the recognition methods are also more traditional based on statistical theory. Finally, the use of data modality is relatively single, and it is still a difficult task to use only a single modality for effective emotion recognition because of the complexity of emotion. Since the interaction between teachers and students in classroom scenarios is mainly discourse, and the emotions contained in the lesson are essential for the whole classroom, this paper conducts a study on emotion recognition in classroom scenarios based on the text in speech and voice based on these two modalities [7]. By collecting the address and text data of teachers and students in the secondary school classroom, we use deep learning technology to explore the emotion recognition method based on the two modalities of classroom speech and classroom text and, finally, achieve the purpose of automatically recognizing the emotion of classroom speakers and judging the whole classroom emotional atmosphere. For students, it can reflect the learning situation through students' emotions and assist teachers in implementing timely teaching interventions, that is, to transform students' emotional states into teachers' decision-making suggestions and eventually help teachers to carry out accurate teaching; for teachers, automatic recognition of teachers' emotions will allow teachers to reflect on their teaching behaviors after class and improve their teaching ability, which can also be used as a basis for evaluating teachers' teaching level [8]. Realizing the overall emotional portrait of the classroom will facilitate macroscopic decision-making, help teachers grasp the overall teaching atmosphere of the school from the students and their levels, effectively promote objective evaluation of the school, and ultimately make suggestions for improvement from the teachers and students' levels to enhance the overall teaching effectiveness of the school.

RETRACTED

## 2. Related Works

Enough research has been done on classroom emotions to analyze the behavior of teachers and students in the classroom, their emotional expressions, and the effect on the school after these expressions. As early as the 1960s, psychologist DE Caigny A began to join in studying categories related to the emotional goals of teaching and learning and proposed an effective system of classifying emotional domains and goals. The foundational value of education is to achieve development rather than growth than a challenge [9]. Therefore, the most appropriate assessment tool for teaching and implementation is not a norm-referenced test but rather a criterion-referenced test and a continuum that needs to be completed for the respondent according to a hierarchy of levels. This idea has profoundly impacted subsequent research on effective teaching and learning. Kumaran et al. later proposed a classification theory of educational goals, which requires a classification system based on emotions [10]. The classification dimensions are mainly reflected in five levels: acceptance, response, value judgment, organization, and characterization of value and value complexes, all of which have specific emotional meanings and sublevels corresponding to the level. Khare and Bajaj believe that the emotional level can be seen as a continuum of hierarchical levels and that describing emotions is not just a way to simply perform [11].

More and more researchers have been conducting in-depth research in speech emotion recognition. As the study progresses, many open-source tools have emerged, the most popular of which is the genuine smile and opener toolkits developed by Ocquaye et al. This toolkit extracts speech features, providing excellent information convenience for many researchers [12]. These tools can automatically mine the acoustic elements of speech signals, high-dimensional statistical features, and underlying features of the voice and automate a portion of the simple operations related to speech processing independently [13]. Due to their convenience, they are used in bulk in many speech-related tasks in engineering fields. After the idea of speech emotion recognition was proposed, many scholars and researchers have conducted much research in this field. Speech emotion features have been continuously improved, but the results harvested by this method in speech emotion recognition have not reached expectations [14]. Many kinds of classifiers can be applied to this field, among which the most widely used in machine learning with good results are the support vector machine (SVM) and the hidden Markov model (HMM). Chao and Dong once applied both models to emotion recognition and obtained a 70.1% of emotion recognition rate. In recent years, artificial intelligence has gradually entered people's lives, deep learning is getting hotter and hotter, and it has emerged strongly in various fields [15]. Deep neural networks, convolutional, and recurrent neural networks are widely used in speech emotion recognition and have achieved good results.

RETRACTED

With the application of deep learning in SER, scholars have increasingly demanded the recognition performance of the model and proposed many deep learning-based SER algorithms [16]. Unlike the traditional methods used for emotion recognition, most current research uses CNN to extract emotion features directly from the speech spectral graph and then input the elements into the classifier due to the great advantage of CNN in feature extraction [17]. Existing research on deep learning-based SER algorithms can be divided into two categories: the first category is CNN structure-based speech emotion recognition algorithms. Maximum pooling is used to extract salient features in the spectrogram. An attention mechanism is further introduced after complete pooling to investigate the effects of different elements, speech signal length, and different types of speech on the performance of emotion recognition [18]. In recent years, CNN has become very popular in the image field, playing an essential role in credit and classification. They belong to a kind of deep learning, which can discover on their own some information that is difficult to be found by humans but easily distinguished by computers and uncovers the hidden contents [19]. The color of each coordinate point corresponds to the strength of speech energy, which reflects the change in the power of the speech signal at different frequencies over time, and contains a lot of information. Based on the speech spectrogram, Hizlisoy et al. applied the SVM classifier to replace the softmax classifier to improve the effect of emotion recognition [20]. Song et al. proposed a speech spectrogram-based emotion recognition method for elderly speech [21]. Hao used the attention mechanism for deep feature extraction of the address spectrogram and applied it to speech emotion recognition [22]. Ying and Yizhe used the DNN network to extract the research of bottleneck features for emotion recognition and have made some progress [23].

## 3. Design of Classroom Emotion Recognition Model Based on Convolutional Neural Network Speech Emotion Algorithm

### 3.1. Convolutional Neural Network Speech Emotion Algorithm Model Construction

Speech emotion recognition algorithms can mainly include machine learning algorithms based on KNN, random forest, SVM, and methods based on deep learning techniques DNN, CNN, and RNN. K nearest neighbor algorithm is a simple classification method based on statistics, widely used in classification algorithms [24]. The core idea is to find the K samples closest to the unknown sample points and determine the class information of the unknown samples from these K samples.

RETRACTED

Given the training dataset *t* = {(*x*_1_, *y*_1_), (*x*_2_, *y*_2_), ⋯, (*x*_*n*_, *y*_*n*_)} and the samples to be tested *x*, the class of the models is calculated, where *x*_*i*_ ∈ *x* are the instance's feature vector, the example's feature vector, and the standard type. According to the given distance criterion, the distance between the sample to be measured and all models in the training set is calculated *d*(*x*, *x*_*I*_), *I* = 1, 2, ⋯, *n*. And find the location of K nearest points to the piece to be measured, denoted as the set *n*_*K*_(*x*). Euclidean distance is the most used metric for measuring distance. The formula can express an example:

(1) $$\begin{array}{c} d\left(x\right)=\overset{n}{\underset{l=1}{\sum }}{\left(x_{i}+x_{l}\right)}^{2}. \end{array}$$

The final category of the sample to be tested *x* is determined in the set *n*_*K*_(*x*) according to some classification difference rule; in the case of the majority table decision rule, the final category *y* can be expressed as an equation.

(2) $$\begin{array}{c} y=\sum \max\sqrt{\left(n_{K^{\left(x\right)}}-1\right)}. \end{array}$$

In the measure of distance, the choice of *K* value size is an essential factor affecting the performance of the KNN algorithm. In machine learning, cross-validation is often used to select the parameters. The dataset is divided into training, validation, and test sets. The model parameters are decided by observing the performance of the model trained on the training set on the validation set. Finally, the final model version is tested on the test set. For example, overfitting problems will quickly occur if the *K* value is too small. The *K* value can be adjusted by observing the model's performance on the validation set to ensure that the model performs optimally on this dataset.

In machine learning, the performance of a single model is often not very satisfactory. It is often combined with multiple weak classifiers through an integrated learning approach to eventually form a classifier with excellent performance. Random forest is a typical algorithm in blended learning. The weak classifier used in the random forest is the decision tree. The decision tree model is a tree structure where each internal node represents an attribute or feature on which to make a judgment output, and each node represents a classification result. The decision tree divides subsets by selecting features through specific rule algorithms until the samples in the subsets are classified into the same class. The commonly used algorithms are ID3, C4.5, and CART algorithms. CART is a conditional probability distribution that outputs a random variable *Y* given a random variable *X*. Unlike the decision trees of ID3 and C4.5, the decision trees created by ID3 and C4.5 can be multinomial, with the fork under each node determined by the type of node feature, so that the node can be divided into three divisions. The decision tree is assumed to be a bifurcated tree with internal node features taking the values of “yes” and “no.” The left branch supports the value “yes,” and the left supports the value “no.” Such a decision tree is equivalent to recursively bifurcating each feature, dividing the input space into a finite number of cells, and predicting the probability distribution over these cells, i.e., outputting the conditional probability distribution given the input conditions. Random forest improves the model's generalization by randomizing the selection of samples and randomizing the selection of division attributes. Firstly, a random sample with put-back on the dataset by bootstrap is used as a training subset of each decision tree, and multiple subsets are used to train the decision trees separately. Then, during the decision trees training, a certain number of randomly selected features are used as the division attributes of the decision trees to build the decision trees. Finally, all the generated decision trees are voted to produce the final classification results.

RETRACTED

The core idea of support vector machines is to find a hyperplane that correctly divides the training dataset and requires that this separated hyperplane's geometric interval be maximized. Suppose that for a two-dimensional linear separable space, the dataset *s* = {(*x*_1_, *y*_1_), (*x*_2_, *y*_2_), ⋯, (*x*_*n*_, *y*_*n*_)} is the feature vectors of the instances, and *i* = 1, 2 ⋯ , *nn* is the number of training samples.

(3) $$\begin{array}{c} \left\{\begin{array}{c} w=\underset{i=1}{\sum }\left(a_{i}-y_{i}-x_{i}\right),\\ m=\sum a_{i}y_{i}. \end{array}\right. \end{array}$$

Convolutional neural networks have excellent ability in speech emotion feature extraction, image recognition, handwritten Chinese character recognition, etc., through different layer structures, mainly using local connectivity and global sharing, consisting of convolutional layer, pooling, and fully connected layer. In speech recognition, it has good translational and dimensional invariance and is good at handling speech features in two-dimensional space with good robustness and operational efficiency. Its network structure diagram is shown in Figure 1. The input of CNN is generally a two-dimensional matrix of speech features. It is mainly used to automatically learn speech emotion features by the backpropagation algorithm and continuously optimize the network parameters. The functions of each layer of the convolutional neural network are as follows.

1. Convolutional layer: the main task of the convolutional layer is to automatically learn the input speech features through the convolutional kernel, map the learned features, pass them to the next layer, and learn higher-level features from them based on the lower-level features known in the previous layer. Assuming that the dimension of the two-dimensional input matrix of speech features is *M* × *N*, the size of the convolutional kernel *W* is *I* × *J*, the bias is *b*, the activation function is *f*, and the output is the speech feature matrix *y* with dimension size *M* × *N*, the convolutional operation of CNN is as follows:

(4) $$\begin{array}{c} y_{m-n}=\overset{j-1}{\underset{j=0}{\sum }}\frac{\left(x_{m+i}-x_{n+j}\right)}{\sqrt{b+1}}. \end{array}$$

Usually, a convolutional layer contains multiple convolutional kernels (kernel) to extract different feature information in the same two-dimensional matrix of speech features, equivalent to people observing one thing simultaneously [25]. Still, the focus is not in the same place, so the information extracted by the convolutional layer is more comprehensive. Meanwhile, after the speech emotion features are entirely removed, the convolutional layer will automatically downscale the feature parameters to conclude. A 5 × 5 two-dimensional speech feature matrix is obtained after convolution operation with a convolution kernel of 3 × 3.

(2) Pooling layer: the pooling layer, also known as the downsampling layer, has the main task of downsampling the speech emotion features learned from the convolutional layer. Since the feature redundancy obtained from the convolutional kernel (kernel) is high, the pooling layer can remove the redundant information or reduce the marginal insensitive intake. Usually, a local window (2 × 2) is defined on the feature matrix extracted from the convolutional layer, and pooling is performed by window sliding, calculated as an equation.

(5) $$\begin{array}{c} a_{j}=\int \left(\sum \left(a_{j}^{l-1}+b_{j}^{l}\right)\right.-l \end{array}$$

(3) Fully connected layer: the fully connected layer is the key algorithm to compute the advanced speech emotion feature sequences extracted from the upper two layers of CNN and classify and recognize them, which can realize the learning and memory of the emotion feature matrix. The fully connected layer consists of many neurons. The neurons are optimized by forwarding and backward propagation algorithms, weights of feature parameters, and bias training to achieve speech emotion feature recognition. Traditional neural network: no theory to point out how many layers (the number of layers has no role). Convolutional networks: more effective feature learning part, deepening the network to be effective
(4) Output layer: the output layer is an essential structure for finalizing the classification. After the whole connection is trained by learning, it outputs a string of counts

Therefore, it is necessary to use the output layer to calculate the probability of these results, which can get the maximum likelihood of a specific category to complete the work of classification. Due to the shared convolution kernel, it can handle high-dimensional data well. Need to manually select features and train good weights, i.e., get good results in feature classification. This paper uses the softmax layer as the output layer for type, which converts each neuron's numerical calculation results in the fully connected layer into a relative normalization between 0 and 1. It gives the predicted category based on the close probability. The computational formula is as follows.

(6) $$\begin{array}{c} S=\overset{k}{\underset{j=1}{\sum }}\frac{\left(e^{j}-e^{i}\right)}{\sqrt{\left(e^{j}+e^{i}\right)}}. \end{array}$$

RETRACTED

### 3.2. Classroom Emotion Recognition Model Design

The primary step in performing speech emotion recognition is to address what emotion is and how to describe and represent it. There are two main models to express human feelings: discrete classification and dimensional. The former of the two approaches is, in essence, a classification problem, and the latter is a regression prediction problem.

First, the discrete emotion description model defines a limited number of the universal emotion labels from all human emotion states, which are independent of each other and are called basic emotions. Other emotions are obtained from different permutations of the basic emotions. The four basic emotions recognized and widely used are happiness, anger, sadness, and neutrality. The six basic emotions proposed are happiness, anger, sadness, surprise, disgust, and fear. Since it is easy to understand and has broad applicability, it is being used in more and more emotion recognition fields.

The dimensional emotion description model, also known as the continuous emotion description model, describes specific emotion attributes as coordinates in a spatial dimension. Each axis corresponds to a particular attribute of emotion [26]. Existing theories of specific emotional states can have corresponding coordinates in emotion space, with the values on each axis indicating the intensity of the corresponding attribute. Researchers have proposed different views on what attributes specific emotions should include, power, similarity, and bipolarity to measure the three-dimensional model of emotion; i.e., various emotional states will correspond to different intensities of expression. Unlike the traditional methods used for emotion recognition, most current research uses CNNs to extract emotion features directly from the speech spectral graph and then input the parts into the classifier due to the great advantage of CNNs in feature extraction. And certain emotions will now exist with similar properties or opposing properties. Nowadays, one of the more mainstream emotion description models is the validity-arousal-dominance (PAD) dimensional emotion description model, whose model is shown in Figure 2.

RETRACTED

The primary interaction between teachers and students in classroom scenarios is in the form of discourse, and judging emotions through the lesson is also one of the most common ways. Therefore, this chapter studies speech emotion recognition using the speech data generated from teacher-student communication in classrooms [27]. At the same time, this chapter also references the effect of classroom speech as a single modality for the later multimodal fusion study and an optimal emotion recognition model structure for speech stream branching. The discrete emotion description model describes emotions into discrete categories, such as happy, angry, sad, etc. There are 6 basic human emotions: happy, angry, surprised, sad, disgusted, and scared. According to the corpus data, the Chinese emotion corpus also basically follows these 6 basic emotion categories, except that disgust is replaced with neutral. This dataset refers to a wide range of human emotions and the actual performance in traditional secondary school classrooms. Finally, it identifies nine categories of emotions: hesitation, anger, silence, tension, doubt, satisfaction, surprise, neutrality, and excitement. Three people jointly labeled the feelings of each speech sample in the dataset, and the principle of minority rule determined the final emotion labels of the pieces. The number of examples in each category of emotions in the dataset is shown in Figure 3.

People can capture each other's emotional changes through speech because the human brain can perceive and understand the information in speech signals. This information can reflect the speaker's emotional state. On the other hand, speech emotion recognition is a computer simulation of the human emotion perception process, which extracts emotion-related features from speech signals and learns the mapping relationship between these features and emotions. The selection of parts is the key to speech processing, and the goodness of features directly affects the accuracy of speech emotion recognition models. Therefore, how to extract compelling speech emotion features is very important. Classroom observation is a teaching research activity that seeks to improve students' learning and promote teachers' professional development by recording, analyzing, and studying the operation of a classroom teaching or some issues. It requires the observer to observe with a clear purpose and with their senses and aids. Listening to a classroom is an activity of careful observation, which is extremely important for understanding and knowledge of the classroom. There are many commonplace problems in the classroom that can be explored and thought about through the conscious observation of the listener. Listening is a meaningful way to improve the quality of teachers and the quality of classroom teaching.

RETRACTED

Rhythmic features: in linguistics, rhythm refers to the components of nonindependent segments (vowels and consonants) in speech, forming linguistic functions such as intonation, tone, repetition, and rhythm. Rhyme can reflect various speaker characteristics, including the speaker's emotional information. The verse does not affect the words and phrases of the speech content, but it does affect the true expressed meaning. Given different rhythmic structures, the same sentence can convey different meanings [28]. Therefore, rhythmic features can somewhat characterize the emotional parts of speech. Spectral features: spectral features are the expression of the correlation between vocal tract shape changes and vocal motion. Herman Levin's first study found that emotion's expression influenced speech frequency distribution and suggested that pitch frequency can be used as an emotional state feature.

Voice quality features: voice quality is a subjective evaluation index of people's speech, used to evaluate speech clarity, cleanliness, and recognition. It is found in the listening and speaking experiments that voice quality is often accompanied by gasping, trilling, choking, etc., when the speaker is emotionally excited, so many researchers have applied voice quality features to the field of speech emotion recognition. Emotion-like feature set: emotion-like feature set is a collection of features designed by experts specifically for emotions. The set includes low-level descriptors (LLDs) and high-level statistics functions (HSFs).

The model is improved from the classical CNN model Le Net by replacing the 5 × 5 convolution in the original network structure with two small 3 × 3 convolution kernels, reducing the number of parameters, and using the dropout technique to reduce the degree of overfitting after the two top pooling layers and between the two top layers. The sigmoid activation function of the original model is prone to oversaturation, and the output is 0 or 1 when the absolute value of the input is significant. Still, the gradient of the sigmoid function is close to 0 at these two places, which is prone to gradient loss and leads to an unexpected termination of training. When the input signal exceeds 0, the output value equals the output value of 1.8. Because of its partially linear characteristic, ReLU does not oversaturate. At the same time, ReLU only requires a threshold to obtain the activation value and does not require complex exponential operations like sigmoid, thus reducing the computational effort of training. Sigmoid and ReLU functions are as follows:

(7) $$\begin{array}{c} f_{\left(t\right)}=\sum W_{f}\frac{h\left(t-1\right)}{\sqrt{U_{f}x\left(t\right)-b_{f}}}, \end{array}$$

(8) $$\begin{array}{c} y_{t}=\sum \max\frac{s_{t}-c}{{Us}_{t}}. \end{array}$$

The KNN and SVM models based on traditional acoustic features perform better than the CNN model based on the speech spectrogram in recognition, especially the SVM, recognizing various emotions and the overall performance. The advantage of KNN is that the model is easy to understand, and you can get good performance by not requiring too much tuning. Trying this algorithm is a good benchmark before considering more advanced techniques. SVM is a small dataset with nonlinear rigorous mathematical logic, high accuracy, and good generalization. In terms of individual emotion recognition, the CNN model performs slightly better than KNN in some indicators of emotions, such as fear and sadness. The model's macro-P, macro-R, macro-F1 values, and recognition rate are comparable to the KNN models, which indicates that the CNN method is feasible to a certain extent. Still, the recognition effect and model performance need to be further enhanced.

RETRACTED

## 4. Analysis of Results

### 4.1. Analysis of Classroom Emotion Recognition Model Based on Convolutional Neural Network Speech Emotion Algorithm

The experimental data for classroom text-based emotion recognition are derived from the classroom emotion recognition dataset. Pretrained language models have pioneered a new paradigm in NLP research. There are two ways to utilize pretrained models; one is feature-based, which is also a common approach in transfer learning, where the word vectors from the pretrained language model are used as features input to the downstream target task; the other is fine-tuning-based, where the pretrained model is trained directly on the pretrained model and fine-tuned for the downstream target task after convergence. The other one is based on fine-tuning, i.e., training directly on the pretrained model and fine-tuning for the downstream target task after convergence without training the network from scratch [29]. Fine-tuning the pretrained model is advanced and effective in many experimental studies. The process of fine-tuning the pretraining model is shown in Figure 4. Fine-tuning the pretraining model generally involves four aspects: the corpus, the encoder, the target task, and the fine-tuning strategy. The canon is the massive unlabeled text data used to pretrain the model. Because of the large amount of data in the corpus, the pretrained model tends to learn the underlying semantic information well, and the learning method is unsupervised. An encoder is a pretrained language model used for text feature encoding and thus text representation. Such models should be chosen to have solid representational power; e.g., the multilayer transformer model in BERT has linguistic reliability and symbolic power. The pretrained models can be downstream to interface with different NLP tasks, such as sequence annotation, classification, and sentence relationship determination. When fine-tuning the pretrained model, we need to specify the target task, design the downstream model, and finally utilize the pretrained model and achieve the target task by fine-tuning. The strategy of fine-tuning refers to the way of fine-tuning. There are two common ways of fine-tuning: the first one is to use the pretraining model as a feature extractor and generally take the results of the last layer or the penultimate layers of the pretraining model as the feature input of the downstream task; the second one is to fine-tune the whole model, i.e., to do end-to-end training of the entire pretraining model and the downstream task model with experimental data. Because the pretraining model has already converged and its parameters have been well optimized, the model's parameters will change less during the optimization process, which is called fine-tuning.

As with the classroom speech emotion recognition experiments, 20% of the classroom text data were randomly selected as the test set for the experiments. The remaining text data were used to train and evaluate the text classification model. The text data used for training was enhanced locally by both near-synonym replacement and noise introduction, just like speech. The evaluation metrics for the classroom text sentiment classification models were also taken as weighted accuracy, unweighted accuracy, and macro-F1 scores for each category. The experimental evaluation method uses the fivefold cross-validation method. Each fold is taken after the model converges, explicitly using the early-stop method with little difference in model training accuracy within 5 generations. Other models were also tested in this part of the experiment to compare the performance of different models on classroom text emotion classification. The pretrained word embedding vector initializes the word representation. It allows the word embedding representation to be fine-tuned and optimized during the training process. Then, a native recurrent neural network model is constructed for classroom text emotion recognition using GRU computational units, text recurrent encoder, or TRE model for short. One of the reasons for choosing the GRU recurrent neural network is that GRU has similar experimental effects compared to LSTM, but it is easier to compute. The second comparison model is the Bert model. The Client-l12 model is replaced with the Bert Chinese pretraining model to investigate the differences between the two pretraining models. The training results of the three models are shown in Figure 5.

RETRACTED

The details of the two models, Xlnet-l12 and Tre, are explored in comparison across classroom text sentiment classes. The method used is still error analysis using confusion matrices, the normalized confusion matrix for the Xlnet-l12 model on the test set, and the confusion matrix for the TRE model on the test set. The Client-l12 model has a solid ability to distinguish between silence, doubt, and neutral text emotion classes. Client-l12 outperforms the TRE model in all emotion classes except for the three classroom text emotions of anger, quiet, and surprise, especially in the two emotion classes of doubt and satisfaction. Both have a recall rate of more than 10% compared to the TRE model. This shows that the Xlnet-l1 model uses pretraining and ranked attention mechanisms to deliver more power than the native recurrent neural network model in characterizing text or in the feature extraction of text. The TRE model has extremely high classification ability for the silent classroom text emotion class, followed by better recognition of neutral. The recall of the TRE model on the two emotion classes of silence and anger is like that of the Xlnet-l12 model and has the same performance. Because of silent emotions in the classroom, their text expressions are often composed of blank or a few words that do not contain vibrant color; they can achieve high accuracy for silent emotions, whether the Xlnet-l12 model with the solid representational ability or the slightly inferior TRE model. For anger and hesitation, comparing the previous recognition using speech and the current recognition using text, we can find that the recall rate of rage and uncertainty has not been improved in each modality. On the one hand, each model cannot learn enough differentiated features due to the insufficient sample size of anger and hesitation classes; on the other hand, the model itself has defects, such as model prediction with bias. The comparison of the scores of Xlnet-l12 and TRE classroom emotion recognition models is shown in Figure 6.

RETRACTED

### 4.2. Classroom Emotion Recognition Model Implementation

There will be many network models in training the network. We aim to get network models with good generalization performance and high recognition accuracy, so only the best prediction model and the fitted model are recorded in the experiment. Validation accuracy is a crucial metric for training model generalization. The best prediction model appears when the validation accuracy reaches the maximum value when training the network. The model fits the experimental data better and performs better in speech emotion recognition prediction. The validation accuracy of the improved trained model reaches 92.35% on Emo-DB, the German Berlin sentiment database. The validation accuracy is improved by 8% compared to the built model. Meanwhile, the loss function curve becomes smooth with slight fluctuation after 80 training cycles, and the final convergence value is 0.47. The training model accuracy is shown in Figure 7.

The accuracy of the CNN-BLSTM-hybrid distributed attention mechanism model in speech emotion recognition is improved by about 1% compared with the CNN-BLSTM multiheaded attention mechanism model, which proves that the proposed hybrid distributed attention model effectively solves the low-rank bottleneck problem of multiheaded attention mechanism and enhances the expression ability of the model; the accuracy of CNN improved BLSTM multiheaded attention mechanism model. The accuracy of the CNN improved BLST. Multiheaded attention mechanism model is enhanced by about 6% compared with the CNN-BLSTM multiheaded attention mechanism model, which proves that the improved BLSTM proposed in this paper extracts the contextual temporal information of the spectral map more comprehensively and enhances the temporal feature vector of speech. The accuracy of the model presented in this paper is higher than that of other models in the ablation experiment, which proves that the two innovations proposed in this paper are effective in speech emotion recognition and can better integrate the advantages of temporal and spatial features of the two models, which verifies the effectiveness of the model in this paper. To show the improvement effect of hybrid distributed attention more intuitively on multiheaded attention mechanism, different head parameters are designed to conduct experiments based on the hybrid neural network + combination distributed attention model and hybrid neural network + multiheaded attention model proposed in this chapter, and WA is used as the evaluation index, and the experimental results are shown in Figure 8.

RETRACTED

By comparison, the method proposed in this paper has dramatically improved the recognition accuracy in the category of happy emotions. It has been enhanced from 39% to at most 56%. At the same time, the model's accuracy in recognizing the other three categories of emotions has also improved slightly. Although the fully convolutional network model is not as accurate as the model with recurrent structure, it has an unparalleled advantage in complexity and computational speed. In some mobile devices and tiny sensors, where the model complexity and computational effort are high, it is not easy to meet the requirements using a recurrent structure. The entire convolutional network shows its advantages. However, the confusion matrix also indicates that our model has room for improvement. The accuracy of emotion recognition is only around 80%, which can be improved theoretically by the production and preprocessing of the classroom speech emotion dataset and the training results of the neural network. Data is often more important for deep learning than algorithms because the quality and quantity of data fundamentally determine how well the model is trained. Therefore, the production of datasets and the preprocessing of data are significant. Since the dataset in this paper exceeds the current publicly available datasets in both the number of speakers and the naturalness of speech, the model in this paper has some generalization ability and can be applied to more classroom contents.

## 5. Conclusion

Classroom observation has always been an essential part of the study of education and teaching. Previously, classroom observations were human-based, and people's subjective judgments were used to evaluate the strengths and weaknesses of a class. The data obtained using a convolutional neural network model will be more objective, and the conclusions obtained from extensive data analysis will be more convincing. The convolutional neural network model saves a lot of workforce and time, and we can get the data quickly without watching a whole class to get the research content more easily. This paper proposes an attention mechanism-based algorithm for emotion recognition of variable-length speech, which focuses on essential features by embedding an attention module. This paper presents a spatiotemporal attention module to assign weights to the address spectrogram features. The convolutional channel attention module pays attention to part of the channel features of the CNN and gives the results. The experimental results show that the proposed method in the paper has a significant improvement in recognition accuracy for each emotion classification compared with that before the model improvement, including a 6.7% improvement in WA accuracy and a 9.1% improvement in UA accuracy. We can get macroscopic data patterns and characteristics through extensive data analysis, which is beneficial for us to grasp the big visible picture and discover the features and shortcomings of emotion teaching.

RETRACTED

By using deep learning to study classroom emotions and training a speech emotion recognition model, we can rapidly recognize and classify classroom emotions for the following research step. A classroom speech emotion dataset is constructed. This dataset can be used as the basis for training and refining the speech emotion recognition algorithm to improve the recognition accuracy of the training model in the future; likewise, the dataset needs to be more. Similarly, the dataset needs to be improved and expanded to improve the accuracy of classroom emotion recognition. Based on the obtained classroom emotion data, this paper provides an analysis method that classifies classrooms according to the proportion of labels and then proposes the characteristics and shortcomings of current classroom emotion teaching according to the number and characteristics of each classroom category.

## Figures and Tables

**Figure 1:** CNN network structure diagram.

**Figure 2:** PAD affective description model.

**Figure 3:** Number of samples for each type of emotion.

**Figure 4:** Pretraining model fine-tuning process.

**Figure 5:** Training results of the three models.

**Figure 6:** Comparison of scores of Xlnet-l12 and TRE classroom emotion recognition model.

**Figure 7:** Training model accuracy.

**Figure 8:** Comparison of experimental results of classroom emotion recognition.

## Data Availability

The data used to support the findings of this study are included within the article.

## References

[1] Christy A., Vaithyasubramanian S., Jesudoss A., Praveena M. D. A. (2020). Multimodal speech emotion recognition and classification using convolutional neural network techniques. *International Journal of Speech Technology*.

[2] Shen X., Shi G., Zhang Y., Weng S. (2022). Wireless volatile organic compound detection for restricted Internet of Things environments based on cataluminescence sensors. *Chemosensors*.

[3] Yadav S. P. (2021). Emotion recognition model based on facial expressions. *Multimedia Tools and Applications*.

RETRACTED

[4] Agarwal G., Om H. (2021). Performance of deer hunting optimization based deep learning algorithm for speech emotion recognition. *Multimedia Tools and Applications*.

[5] Shen X., Shi G., Ren H., Zhang W. (2022). Biomimetic vision for zoom object detection based on improved vertical grid number YOLO algorithm. *Frontiers in Bioengineering and Biotechnology*.

[6] Zvarevashe K., Olugbara O. O. (2020). Recognition of speech emotion using custom 2D-convolution neural network deep learning algorithm. *Intelligent Data Analysis*.

[7] Daneshfar F., Kabudian S. J. (2020). Speech emotion recognition using discriminative dimension reduction by employing a modified quantum-behaved particle swarm optimization algorithm. *Multimedia Tools and Applications*.

[8] Abdullah S. M. S., Abdulazeez A. M. (2021). Facial expression recognition based on deep learning convolution neural network: a review. *Journal of Soft Computing and Data Mining*.

[9] De Caigny A., Coussement K., De Bock K. W., Lessmann S. (2020). Incorporating textual information in customer churn prediction models based on a convolutional neural network. *International Journal of Forecasting*.

[10] Kumaran U., Radha Rammohan S., Nagarajan S. M., Prathik A. (2021). Fusion of mel and gammatone frequency cepstral coefficients for speech emotion recognition using deep C-RNN. *International Journal of Speech Technology*.

[11] Khare S. K., Bajaj V. (2020). Time–frequency representation and convolutional neural network-based emotion recognition. *IEEE Transactions on Neural Networks and Learning Systems*.

[12] Ocquaye E. N. N., Mao Q., Xue Y., Song H. (2021). Cross lingual speech emotion recognition via triple attentive asymmetric convolutional neural network. *International Journal of Intelligent Systems*.

[13] Xiao Y., Zhao H., Li T. (2020). Learning class-aligned and generalized domain-invariant representations for speech emotion recognition. *IEEE Transactions on Emerging Topics in Computational Intelligence*.

[14] Yadav S. P., Zaidi S., Mishra A., Yadav V. (2022). Survey on machine learning in speech emotion recognition and vision systems using a recurrent neural network (RNN). *Archives of Computational Methods in Engineering*.

[15] Chao H., Dong L. (2021). Emotion recognition using three-dimensional feature and convolutional neural network from multichannel EEG signals. *IEEE Sensors Journal*.

[16] Chen X., Xie H. (2020). A structural topic modeling-based bibliometric study of sentiment analysis literature. *Cognitive Computation*.

[17] Zhang H. (2020). Research on spoken English analysis model based on transfer learning and machine learning algorithms. *Journal of Intelligent & Fuzzy Systems*.

RETRACTED

[18] Wang C., Ren Y., Zhang N., Cui F., Luo S. (2022). Speech emotion recognition based on multi-feature and multi-lingual fusion. *Multimedia Tools and Applications*.

[19] Ashwin T. S., Guddeti R. M. R. (2020). Automatic detection of students’ affective states in classroom environment using hybrid convolutional neural networks. *Education and Information Technologies*.

[20] Hizlisoy S., Yildirim S., Tufekci Z. (2021). Music emotion recognition using convolutional long short term memory deep neural networks. *Engineering Science and Technology, an International Journal*.

[21] Song P., Zheng W., Yu Y., Ou S. (2021). Speech emotion recognition based on robust discriminative sparse regression. *IEEE Transactions on Cognitive and Developmental Systems*.

[22] Hao K. (2020). Multimedia English teaching analysis based on deep learning speech enhancement algorithm and robust expression positioning. *Journal of Intelligent & Fuzzy Systems*.

[23] Ying X., Yizhe Z. Design of speech emotion recognition algorithm based on deep learning.

[24] Mihalache S., Burileanu D. (2021). Dimensional models for continuous-to-discrete affect mapping in speech emotion recognition. *University Politehnica of Bucharest Scientific Bulletin, Series C*.

[25] Zatarain Cabada R., Rodriguez Rangel H., Barron Estrada M. L., Cardenas Lopez H. M. (2020). Hyperparameter optimization in CNN for learning-centered emotion recognition for intelligent tutoring systems. *Soft Computing*.

[26] Takalkar M. A., Xu M., Chaczko Z. (2020). Manifold feature integration for micro-expression recognition. *Multimedia Systems*.

[27] Saurav S., Gidde P., Saini R., Singh S. (2022). Dual integrated convolutional neural network for real-time facial expression recognition in the wild. *The Visual Computer*.

[28] Patel N., Patel S., Mankad S. H. (2022). Impact of autoencoder based compact representation on emotion detection from audio. *Journal of Ambient Intelligence and Humanized Computing*.

[29] Mungra D., Agrawal A., Sharma P., Tanwar S., Obaidat M. S. (2020). PRATIT: a CNN-based emotion recognition system using histogram equalization and data augmentation. *Multimedia Tools and Applications*.

